This article has been retracted.

# Chemopreventive Evaluation of a Schiff Base Derived Copper (II) Complex against Azoxymethane-Induced Colorectal Cancer in Rats

**DOI:** 10.1371/journal.pone.0091246

**Published:** 2014-03-11

**Authors:** Maryam Hajrezaie, Pouya Hassandarvish, Soheil Zorofchian Moghadamtousi, Nura Suleiman Gwaram, Shahram Golbabapour, Abdrabuh NajiHussien, Amel Abdullah Almagrami, Maryam Zahedifard, Elham Rouhollahi, Hamed Karimian, Somaye Fani, Behnam Kamalidehghan, Nazia Abdul Majid, Hapipah Mohd Ali, Mahmood Ameen Abdulla

**Affiliations:** 1 Department of Biomedical Science, Faculty of Medicine, University of Malaya, Kuala Lumpur, Malaysia; 2 Institute of Biological Sciences, Faculty of Science, University of Malaya, Kuala Lumpur, Malaysia; 3 Department of Chemistry, University of Malaya, Kuala Lumpur, Malaysia; 4 Department of Pharmacy, Faculty of Medicine, University of Malaya, Kuala Lumpur, Malaysia; Faculty of Pharmacy, Ain Shams University, Egypt

## Abstract

**Background:**

Based on the potential of Schiff base compounds to act as sources for the development of cancer chemotherapeutic agents, this *in vivo* study was performed to investigate the inhibitory properties of the synthetic Schiff base compound Cu(BrHAP)_2_ on colonic aberrant crypt foci (ACF).

**Methodology:**

This study involved five groups of male rats. The negative control group was injected with normal saline once a week for 2 weeks and fed 10% Tween 20 for 10 weeks, the cancer control group was subcutaneously injected with 15 mg/kg azoxymethane once per week for two consecutive weeks, the positive control group was injected with 15 mg/kg azoxymethane once per week for two consecutive weeks and 35 mg/kg 5-fluorouracil (injected intra-peritoneally) for 4 weeks, and the experimental groups were first injected with 15 mg/kg azoxymethane once per week for two consecutive weeks and then fed 2.5 or 5 mg/kg of the Schiff base compound once a day for 10 weeks. Application of the Schiff base compound suppressed total colonic ACF formation by up to 72% to 74% (*P*<0.05) when compared with the cancer control group. Analysis of colorectal specimens revealed that treatments with the Schiff base compound decreased the mean crypt scores in azoxymethane-treated rats. Significant elevations of superoxide dismutase, glutathione peroxidase and catalase activities and a reduction in the level of malondialdehyde were also observed. Histologically, all treatment groups exhibited significant decreases in dysplasia compared to the cancer control group (*P*<0.05). Immunohistochemical staining demonstrated down-regulation of the PCNA protein. Comparative western blot analysis revealed that COX-2 and Bcl2 were up-regulated and Bax was down-regulated compared with the AOM control group.

**Conclusion:**

The current study demonstrated that the Cu(BrHAP)_2_ compound has promising chemoprotective activities that are evidenced by significant decreases in the numbers of ACFs in azoxymethane-induced colon cancer.

## Introduction

Colorectal cancer, also known as large bowel cancer, can involve aberrant growths in the appendix, colon and rectum and is among the three most prevalent types of cancer [1]. Despite much research and progress on the prevention and treatment of colon cancer, significant suppression of tumors is still rarely achieved, and treatment with known agents can lead to tumor progression in some cases [2]. The detection and treatment of early-stage colon cancer with proper agents plays a critical role in reducing the number of colorectal cancer victims [3]. The azoxymethane (AOM) model of experimental colon cancer imitates the extensive molecular, clinical and histological features of human colon cancer [4]. The azoxymethane (methyl-methylimino-oxidoazanium) compound is an oxide of azomethane (molecular formula C_2_H_6_N_2_O) and is commonly used to induce colon cancer in experimental models [5], [6].

Metal complexes have been extensively used in pharmacology for centuries [7], [8]. The development of metal-based drugs has been promoted by significant accomplishments that have been achieved with platinum-based antitumor agents, such as oxaliplatin, cisplatin and carboplatin. However treatment with platinum-based drugs is normally associated with the evolution of drug resistance and severe side effects during the therapy processes [9]. Copper is well known to be a vital cation for cell survival, which plays an essential role as a cofactor of some metalloenzymes. Copper has been an excellent candidate for cancer treatment since the 1960s [10]. The oxidative nature and bio-activity of copper in humans has attracted inorganic chemists to address the pharmacological applications of copper (II) [11], [12]. These types of metals with the unique character of reactivation with dioxygen are used in the body system after passing through the intestinal walls [13]. Because of their potential for DNA cleavage via oxidative or hydrolytic mechanisms and strong interactions with DNA via intercalation or surface associations, copper (II) complexes with heterocyclic bases have been widely investigated [14]. Schiff bases are a notable class of compounds with significant potential anti-ulcer [15], antibacterial, antifungal [16], [17], anti-diabetic [18], antitumor [19]–[23], anti-proliferative [24], [25] and anti-inflammatory activities [26], [27].

Schiff base-derived copper (II) complexes have strong anti-proliferative, gastroprotective and antibacterial potential because of the properties of their metal centers or their coordinate ligands, which are associated with electronic and structural characterizations that are attributable to their coordination [15]. The present study was designed to investigate the inhibitory effect of a copper (II) complex derived from N,N'-dimethyl ethylene diamine and the 2-hydroxyacetophenone Schiff base ligand Cu(BrHAP)_2_ against AOM-induced colon carcinogenesis in rats in terms of the incidence of ACF.

## Materials and Methods

### Chemicals

For this experiment, the carcinogenic chemical of azoxymethane (AOM) was purchased from Sigma Aldrich (St. Louis, MO, USA), and 5-fluorouracil, a colon cancer positive reference, was purchased from Calbiochem (San Diego, CA, USA).

### Synthesis of the complex

The copper complex was synthesized as previously detailed in a published article [15]. This Cu(BrHAP)_2_ Schiff base compound was attained from the Chemistry Department of the Faculty of Science of the University of Malaya.

### Ethical issues

The protocol for this study was approved by the ethics committee for animal experimentation of the Faculty of Medicine, University of Malaya, Malaysia (Ethic No. PM/27/07/2010/MAA (R)). The animals were cared for according to the criteria of the National Academy of Science's Guide for the Care and Use of Laboratory Animals [28], [29].

### Acute toxicity evaluation

To demonstrate the safety of the usage of the Cu(BrHAP)_2_ complex, 36 healthy female and male rats (weighed between 150–180 g) taken from the Animal House of the Faculty of Medicine of the University of Malaya, Kuala Lumpur, underwent acute toxicity analysis. The rats were divided into the following three groups: a vehicle control group, a group that received 100 mg/kg copper (II) complex, and a group that received 2000 mg/kg copper (II) complex [15]. After an overnight fast, the rats were fed the copper (II) complex and were subsequently observed every two hours over 24 hours, and any toxicity symptoms were recorded. Mortality was recorded over the 14 days of the experiment. After the rats were sacrificed, the blood and organs were collected for biochemical, hematological and histological analyses.

### Assessing the chemopreventive effect of copper (II) complex

Male Sprague-Dawley rats were obtained from the Animal House of the Faculty of Medicine, University of Malaya. International principles and local regulations were observed regarding the care and use of these laboratory animals. The rats weighted approximately 180–200 grams and were received at the approximate age of 6–8 weeks. The animals were maintained under controlled conditions at room temperature (22–24°C) and 50–60% humidity on a 12 hr light-dark cycle with ad libitum access to standard diet and water. The animals were acclimatized to the standard laboratory conditions for a period of two weeks before the initiation of any experiment.

Thirty-six adult male rats were divided randomly into the following five groups of six rats each: a negative control group (these rats were received subcutaneous injections of normal saline and were orally administered 10% Tween 20 each day for 10 weeks), a cancer control group (these rats received subcutaneous injections of 15 mg/kg AOM once per week for two consecutive weeks. They were administered orally with 10% Tween 20 (5 mL/kg) daily), a positive control group (these rats received subcutaneous injections of 15 mg/kg AOM once per week for two consecutive weeks and followed with intra-peritoneal injections of 35 mg/kg 5-fluorouracil for 4 weeks) and two treatment groups (these rats first received subcutaneous injections of 15 mg/kg AOM once per week for two consecutive weeks and oral administration of the Cu(BrHAP)_2_ Schiff base compound at dosages of 2.5 mg/kg or 5 mg/kg for 10 weeks) [5]. During the experiments, the rats were weighed and observed daily for signs of toxicity.

### Scoring of aberrant crypts

To record the incidence of ACF, the locations and numbers of crypts were recorded 10 weeks after the last AOM injection. To do this, the rats were killed with a high dose of xylazine and ketamine anesthesia, and their colons were extracted and flushed with cold phosphate-buffered saline (PBS) and then longitudinally opened from anus to rectum. For topographic analysis, 0.2% methylene blue was used to stain the colon, and the colon was observed mucosal side up with a Nikon dissecting microscope. The ACF score was calculated based on the number of aberrant crypts foci, which are known as foci containing more than two aberrant crypts. The number of ACF per colon and the number of aberrant crypts in each focus were determined.

### Histological classification of ACFs

Buffered formalin (10%) was used to fix the colon specimens following processing in a paraffin tissue-processing machine (Leica, Germany). The tissues were then embedded in paraffin blocks and cut into 5-μm sections. The sections were stained with hematoxylin and eosin (H&E) and were observed with a light microscope (Nikon, Japan).

### Immunohistochemistry

After heating the tissue section slides in a hot-air oven for 25 min at 60°C, xylene and alcohol were used to de-paraffinize and rehydrate the tissue, respectively, which was then immunohistochemically stained according to the manufacturer's protocol (Dakocytomation, USA). A peroxidase block was used to block endogenous peroxidase (0.03% hydrogen peroxide-containing sodium azide) and after washing with washing buffer, the slides were incubated with diluted mouse PCNA (1∶200, Cat: ab2426) monoclonal antibody, which was provided by the Abcam Company. Sufficient amounts of streptavidin–HRP were incubated with the sections for 15 min. After washing gently with washing buffer, the sections were incubated with DAB-substrate-chromagen for 5 min and then stained with hematoxylin for 5 sec. They were then dipped in ammonia 10 times and washed with distilled water, and the slides were mounted with a cover slip. Positive samples displayed a brown color under a light microscope. The PCNA labeling index (PI) was measured as the [(number of positive cells)/(total number of epithelial cells)] X 100 for each field. These PI values for all the different colon sections of the rats belonging to similar groups were then averaged.

### Western Blot analyses

After sacrificing the rats, the colon tissue was collected, and to analyze protein expression through western blot analysis, proteins were extracted using protein extraction buffer (Pierce, USA), and the supernatant was subjected to western blot assays.

In brief, extracted proteins (30 μg) were separated on 10% resolving polyacrylamide gels (i.e., SDS-PAGE) and electroblotted (25 mA for 2 h). Extracted proteins were transferred to PVDF membranes (Pierce, USA) using a Trans-Blot SD semi-dry transfer cell (Bio-Rad, USA) at 15 V, 95 mA, for 1 h then the PVDF membrane was blocked using Blocker Casein (Pierce, USA) for 1 h at room temperature and washed twice using TBST. After incubation overnight at room temperature with specific primary antibodies (β-actin 1∶10000 (Cat: ab6276), Bax 1∶1000 (Cat: ab7977), Bcl-2 1∶1000 (Cat: ab183656) and COX-2 1∶1000 (Cat: ab15191), the blots were incubated for 2 h with the appropriate peroxidase-coupled secondary antibodies, and subsequent detection was performed with XOMAT film via enhanced chemiluminescence. The xerograms were digitized with an Epson scanner, and band intensities were quantified using IP lab gel.

### Antioxidant activities of colon homogenates

After washing the colon tissue samples with ice-cold saline, a homogenate (10% w/v) was prepared in ice-cold 50 mM phosphate buffer (pH 7.4) containing a mammalian protease inhibitor cocktail and centrifuged at 10,000×g for 30 minutes at 4°C. Next, the supernatant was used to analyze the activities of the catalase (CAT), glutathione peroxidase (GPX), and superoxide dismutase (SOD) enzymes and for MDA assay. The kits were provided by Cayman Chemical Co. (Michigan, USA).

### Statistical analyses

Predictive Analysis Software (PASW) version 18 was used to analyze the data of this study. The experimental data were analyzed with one-way analyses of variance (ANOVAs) followed by Tukey's post-hoc test. The data are displayed as the means ± the (standard error of the mean) S.E.M. The level of significance was set at *P*<0.05.

## Results

### Acute toxicity study

As reported in our previously published article, the application of the copper (II) Schiff base compound produced no signs of hematology, serum biochemical abnormality, or hepatic or renal toxicity. Thus, this complex seems to be safe for use [13].

### Body weights and serum biochemistry analyses of the chemopreventive potential of the Cu(BrHAP)_2_

No significant differences were observed in the rats' body weights across groups (Table 1). Tables 2 and 3 illustrate the serum biochemistry analyses of the blood collected from the scarified animals for the examination of the parameters of liver and renal function compared to their vehicle groups.

**Table 1:** Effects of the copper (II) complex on body weights in AOM-induced colon cancer.

Groups	Week 1	Week 2
**Negative Control group**	150.2±3.8	355.6±10.6
**Cancer Control group**	149.8±5.7	379±15.8
**Positive Control group**	152.8±4.2	360.7±12.3
**Cu(BrHAP)_2_(2.5 mg/kg)**	151.1±4.5	375.8±20.3
**Cu(BrHAP)_2_ (5 mg/kg)**	153.4±6.3	368.4±9.9

The values are expressed as the mean ± the S.E.M. There were no statistically significant differences between the groups. *P*<0.05 was considered to be significant.

**Table 2:** Effects of the copper (II) complex on parameters of renal function in AOM-induced colon cancer.

Group	Urea (mmol/L)	Creatinine (μmol/L)
**Negative control group**	5.55±0.20	54.5±5.32
**Cancer control group**	5.95±0.06	33.0±2.2
**Positive control group**	5.1±0.42	44.0±0.63
**Cu(BrHAP)_2_(2.5 mg/kg)**	5.5±0.46	33.5±0.57
**Cu(BrHAP)_2_ (5 mg/kg)**	5.3±0.82	33.9±0.89

The values are expressed as the mean ± the S.E.M. There were no statistically significant differences between the groups. *P*<0.05 compared to cancer control group was considered to be significant.

**Table 3:** Effects of the copper (II) complex on liver function in AOM-induced colon cancer.

Groups	Total protein (g/L)	Albumin (g/L)	AST (IU/L)	ALT (IU/L)	GGT(IU/L)
**Negative control group**	67.32±0.34	12.27±0.54	207.2±2.53	63±2.38	5.5±0.3
**Cancer control group**	69.5±0.39	9.0±0.31	229.6±7.2	69.5±0.68	3.7±0.6
**Positive control group**	73.6±2.1	11.3±0.89	182.0±4.5	50.0±0.92	6.1±0.48
**Cu(BrHAP)_2_ (2.5 mg/kg)**	68.5±0.67	10.5±0.4	209.5±6.1	64.2±0.63	4.1±0.1
**Cu(BrHAP)_2_ (5 mg/kg)**	70.9±1.1	11.3±0.42	212.0±10.6	62.0±3.4	4.3±0.32

The values are expressed as the mean ± the SEM There were no significant differences between groups. The significance value was set at P < 0.05 compared to the cancer control group. TB: total bilirubin; ALT: alanine aminotransferase; AST: aspartate aminotransferase; GGT: g-glutamyl transferase.

### ACF frequency

The tumor quantification analyses of the colons that were stained with methylene blue immediately after sacrifice are summarized in Table 4. Figure S1 displays topographic views of the methylene blue-stained colon tissues of the different groups. ACFs were distinguished from the surrounding normal crypts by their increased sizes, the increased distances from the lamina to the basal surfaces of the cells, and the easily discernible pericryptal zones. No microscopic changes were observed in the normal control group, and a significantly greater number of ACFs were recorded in the cancer control group. The groups that received the copper (II) complex exhibited significant reductions in ACF numbers (72.2% and 74.7%; *p*<0.05). The distribution of ACFs in the cancer control group was centered on the middle of the colon in the cancer control group, and the copper (II) complex-treated groups exhibited significantly reduced distal, middle and proximal ACF distributions compared to the cancer control group (Table 5).

**Table 4:** Effects of the copper (II) complex on AOM-induced colonic ACFs containing four or more aberrant crypts.

Treatment group	No. of crypts per ACF				Total ACF	Inhibition %
	1 crypt	2 crypt	3 crypt	4 crypt and more		
**Negative control group**	0.0	0.0	0.0	0.0	0.0	0.0
**Cancer control group**	5±0.43	26±3.27	19±3.27	29±1.27	79±6.7	0
**Positive control group**	1±0.03*	5±0.69*	4±0.64*	8±0.26*	18±2.81*	77.2*
**Cu(BrHAP)_2_ (2.5 mg/kg)**	6±0.71*	5±0.14*	2±0.19*	10±1.04*	22±2.70*	72.2*
**Cu(BrHAP)_2_ (5 mg/kg)**	2±0.41*	4±0.52*	3±0.27*	11±1.13*	20±1.53*	74.7*

The values are expressed as the mean ± the S.E.M. The significance value was set at P< 0.05 compared to the cancer control group.

**Table 5:** Effects of the copper (II) complex on the regional distribution of colonic ACF in AOM-induced colonic cancer.

Groups		ACF Counting		Total
	Proximal	Middle	Distal	
**Negative control group**	0.0	0.0	0.0	0.0
**Cancer control group**	25±3.66	43±5.77	11±3.79	79±6.7
**Positive control group**	0 00±0.0*	18±2.37*	0 00±0.0*	18±2.81*
**Cu(BrHAP)_2_ (2.5 mg/kg)**	7±1.04*	13±7.89*	2±0.5*	22±2.70*
**Cu(BrHAP)_2_ (5 mg/kg)**	0 00±0.0*	20±4.84*	0±0.0*	20±1.53*

The values are expressed as the mean ± the S.E.M. The significance value was set at P< 0.05 compared to the cancer control group.

### Histological evaluation

The macroscopic pathological differences in the colon tissues of different groups indicated that the ACFs contained narrow luminal epithelial cells and deformed goblet cells with elongated nuclei. Losses of cell polarity and increases in mitoses were also observed in dysplastic ACFs compared to the normal circular-shaped cells with basally located nuclei. Histological photos of the colon tissues from the positive control group exhibited reductions in the numbers of cells with pathological differences, and a similar reduction was observed in the oral copper (II) complex treatment groups (Figure S2).

### Immunohistochemistry

Immunohistochemical PCNA protein staining of the colon sections from the azoxymethane group revealed an up-regulation of the protein. The positive control group exhibited a lower number of positive cells compared to the azoxymethane group, and similar results were observed in the copper (II) complex treated groups. The PCNA-positive cells (%) of the colon tissue in the cancer control group were 100%, whereas PCNA-positive cells (%) from the treated group were 47.4% and 35.4%, respectively (*p*<0.05) (Figure 1).

**Figure 1:** Immunohistochemical analyses of the expression of PCNA in the colon tissues. A) Normal colon mucosa. B) Colon mucosa of the group exposed to AOM. C) Colon mucosa of the group treated with 5-fluorouracil. D) Colon mucosa of the group treated with 2.5 mg/kg copper (II) complex. E) Colon mucosa of the group treated with 5 mg/kg copper (II) complex. Immunohistochemical staining for PCNA protein revealed a down-regulation of PCNA protein in the rats treated with the Cu(BrHAP)_2_ complex. Magnification: 100x. All values are expressed as the means ± the standard error of mean. The mean difference was significant at the p<0.05 level compared to the cancer control group.

### Western blot analyses

Western blot analyses revealed that the Bax (23 kDa) protein was down-regulated in the cancer control group and that the Cu(BrHAP)_2_ complex increased the expression of this protein. The Cu(BrHAP)_2_ complex and 5-fluorouracil caused down-regulations of COX-2 (69 kDa) and Bcl2 (26 kDa) proteins in the treated rats compared to the cancer control group. Protein expressions from western blots were quantitated using the Image J software program. The densities for the cancer group (A) were set to 1 and the relative densities for the positive and treated groups were plotted. The data are the mean ± SEM. Statistical significance was expressed as p<0.05 (Figure 2).

**Figure 2:** Western blot analyses of Bax, Bcl-2 and COX-2. A) Colon mucosa of the group exposed to AOM. B) Colon mucosa of the group treated with 5-fluorouracil. C) Colon mucosa of the group treated with 2.5 mg/kg copper (II) complex. D) Colon mucosa of the group treated with 5 mg/kg copper (II) complex. COX-2 and Bcl2 expression was increased and Bax expression was decreased in the treatment group compared to the AOM control group. β-actin was used as an internal control to confirm equal sample loading. The Image J program was used to evaluate protein expression. All values are expressed as the means ± the standard error of mean. The mean difference was significant at the p<0.05 level compared to the cancer control group.

### Antioxidant enzyme activities

The Cu(BrHAP)_2_ complex significantly increased the levels of SOD, CAT and GPX in homogenized colon samples compared to those of the cancer control group (*p*<0.05). The level of MDA was significantly decreased in the Schiff base complex-treated groups, and the cancer control group exhibited an up-regulation of the expression level of MDA (*p*<0.05) (Figure 3).

**Figure 3:** Effects of the copper (II) complex on antioxidant enzyme activities. A) Negative colon group, B) group exposed to AOM, C) group treated with 5-fluorouracil, D) group treated with 2.5 mg/kg copper (II) complex, E) group treated with 5 mg/kg copper (II) complex. All values are expressed as the means ± the standard error of mean. The mean difference was significant at p<0.05 compared to the cancer control group.

## Discussion

Anticancer drug discovery based on biological strategies of using transitional metal chemistry to target cancer growth pathways and activate cancer cell apoptosis have been developed to decrease the severity of cancer in patients [30], [31].

According to recent research that suggests that to control cancer growth, it is not enough to rely on a single cellular or physiological event, looking for the agents with a controlling role in multiple tumorigenic events and associated mechanisms is extremely important [32], [33]. Schiff base groups of compounds have been extensively studied for their chemoprotective effects. The copper complex has the ability to inhibit cells' activities relevant to cell proliferation, and thus deduce the proliferation markers and the elevation of apoptosis pathways [10], [15]. The previous studies reported that proteasome inhibitors induce apoptosis and have potential anticarcinogenic roles [34], [35]. A study by Xiao *et al*. [36] revealed the inhibitory role of Schiff base copper against proteosome activity, allowing the induction of apoptosis to increase.

In the present study, we demonstrated that Cu(BrHAP)_2_ can reduce ACF formation and therefore colon tumor incidence in rats. Mechanistically, the compound showed promising chemopreventive effects against ACF formation by inhibiting tumor cell proliferation and controlled the expression of specific key proteins and mitochondrial apoptosis induction. It appears that controlling the antioxidant enzymes' expression levels with the compound plays an important role in inhibiting ACF formation (Figures 1, 2, 3).

When animal models are used in the study, clinical and toxicological investigations of new synthetic compounds are crucial for ensuring the safety and efficacy of these compounds. As reported in our previously published article, the LD_50_ of Cu(BrHAP)_2_ observed in this study can be considered to be safe based on the global harmonized system of the classification and labeling of chemicals [15], [28]. Thus, our results demonstrated the toxicological safety of the oral administration of this compound because there were no signs of behavioral abnormalities or weight loss. No significant differences were found in the treated groups compared to the control group in terms of liver and renal function. Thus, our findings support the logical use of this new synthetic Schiff base compound.

The carcinogenic compound dimethyl diazene-1-oxide (azoxymethane) has been proven to be capable of producing colon tumors after administration to male rats for a specified period of time [37]. The sizes and numbers of aberrant crypt foci are used as intermediate biomarkers and correlate with the risk of developing colon cancer. Thus, sizes and numbers of aberrant crypt foci provide a quick measure for screening compounds that might be effective in suppressing the development of colon cancer [38]–[40]. As explained previously, through the induction of apoptosis activation via the mitochondrial pathway, the copper complex has the ability to prevent cancers [10]. The present study revealed that the administration of Cu(BrHAP)_2_ at doses of 2.5 mg/kg and 5 mg/kg significantly reduced total AOM-induced colonic ACF formation and multicrypt aberrant crypt growth by 72% and 74% (*p*<0.05), respectively.

The presence of PCNA was used as a marker of cell proliferation (which plays an important role in cancer progression) in the colon tissues because PCNA indicates a cell's extra division capability [41]–[43]. Studies in animal models showed that abnormal epithelial cell proliferation is one of the earliest indications of pre-neoplasia [44]–[45]. Based on a study by Deschner EE *et al*. [46], animals treated with any chemical colon carcinogen revealed a larger proliferation zone and a higher labeling index compared with the vehicle-treated group. According to the immunohistochemical results of this investigation, Cu(BrHAP)_2_ induced colon tissue protection by down-regulating PCNA. Therefore, the groups treated with the compound had a smaller proliferation zone and a lower labeling index, so the cells were no longer in the growth cycle (*p*<0.05). A similar reduction in proliferating cell nuclear antigen was reported previously in a study that demonstrated successful chemoprevention against AOM-induced colon cancer in an animal model [47]. Thus, the compound used in this experiment may inhibit ACF formation by modifying cell proliferation. Multiple factors in the immune apoptosis pathway play critical roles in the survival or death of cells, and these factors interact to affect the final outcomes [47]. The induction of colon cancer with AOM causes oxidative injuries following lipid peroxidation production in colon cells and erythrocytes, which cause increased secretion of total protein and albumin via the kidney, which, in turn, results in the elevation of urea concentrations in the blood. This process may play a role in the etiology of colon cancer in rats [48]–[49] The balance between the ROS levels in the body is essential for cellular function and the apoptotic pathway in precancerous cells [50]. If there is no effective regulation, the excess ROS would damage proteins, lipids or DNA and in turn inhibit the normal function and modulation of gene expression, cell cycle, cell metabolism, cell adhesion and cell death [51]. The Schiff based compound used in this study is presumed to have the ability to counterbalance these ROSs. The mechanism of action of this compound might be through free radical scavenging and quenching of the formation of singlet oxygen, which protects the colon against oxidative stress and stimulated colon repair mechanisms. There is a possibility that the compound possesses protective effects against ACF formation and colon injury through the endogenous oxidative enzyme systems involved in the colon defense system, such as (CAT), (SOD) and (GPX), which counterbalance the oxidative stress induced by AOM. In this study, it was demonstrated that AOM administration caused severe damage to the rat's endogenous antioxidant system, represented by the disturbance of oxidative stress enzymes (CAT, SOD and GPX) activities which led to a decrease in their levels, alongside lipid peroxidation that was characterized by up-regulation in MDA levels.

Previous studies have proven the role of the increased activities of antioxidant enzymes (SOD, CAT and GPX), which are induced by antitumor agents, in the mechanism of chemopreventive therapy [52]. The *in vivo* evaluation of antioxidants performed in this study demonstrated significant elevations in the SOD, CAT and GPX activities in the groups treated with Cu(BrHAP)_2_. However, reduced lipid peroxidation suggested a significant decrease in MDA levels. Although this result was not significant due to the effect of Cu(BrHAP)_2_ on the neutralization of the toxic compounds that are produced by converting AOM to a highly toxic metabolite, the levels of total protein, albumin and urea were restored to normal values [53]. To further investigate the chemopreventive activity of this compound in colon cancer and the mechanism underlying this effect, the expressions of Bax, proapoptotic proteins, B-cell lymphoma 2 (Bcl-2) (which has antiapoptotic effects) and cyclooxygenase 2 (COX-2) in the different groups were analyzed. Western blot assay was used in this study to detect specific proteins in the homogenized extracted colon. These proteins play essential roles in the development of new cancer drugs [54]. Bcl-2 plays a vital role in controlling the process of cell death by blocking various apoptosis signals. In contrast, the Bax protein has a role in the release of a factor that promotes apoptosis into the cytoplasm. Thus, the balance of the expressions of Bcl-2 and Bax is important in the process of cell death [52]–[55]. COX-2 has been reported to be overexpressed in the early stage, and COX-2 levels have been reported to increase with the progression of cancer. COX-2 is the rate-limiting enzyme in the biosynthesis of prostanoids, which increase proliferation, apoptotic resistance and angiogenesis during colonic carcinogenesis. The expression of COX-2 was upregulated in the AOM-induced colonic tumors. Down-regulation of COX-2 has been demonstrated to have a crucial role in the anticancer agent-induced suppression of AOM-induced tumorigenesis in an animal model [53]. Our results revealed that Cu(BrHAP)_2_ increased the expression of the BAX protein, which is inconsistent with a previous study by Zhang *et al*. [56] who reported that the induction of BAX protein expression led to cell apoptosis using Schiff base copper compound, and down-regulated the expression of COX-2 and Bcl-2 proteins, and this pattern of expression changes strongly suggests that apoptosis will be induced via the mitochondrial pathway. Ma *et al*. [10] also demonstrated the anti-cancer effect of a novel Schiff base copper (II) complex through the activation of the mitochondrial pathway. The result of this study was similar with our previous published research on the same compound, which revealed its effective role on gastro-prevention. The result demonstrated that the complex was able to significantly reduce the Bax protein expression [15]. Previous evaluations of effective chemopreventive agents have also revealed the same pattern of Bax, Bcl-2, and COX-2 protein expression [52], [53].

## Conclusions

Based on the result of this study, the chemopreventive potential of Cu(BrHAP)_2_ was demonstrated by reductions in the numbers of ACFs which could be attributed to the down-regulation of cell proliferation-promoting proteins in cancer cells and the elevation of the levels of antioxidant enzymes. Western blot analyses revealed that the copper (II) complex activated apoptosis via the mitochondrial pathway by down-regulating COX-2 and Bcl-2 and up-regulating Bax.

## Supporting Information

Figure S1 **Topographical views of colon mucosa.** A) Normal colon mucosa. B) Colon mucosa of the group exposed to AOM. C) Colon mucosa of the group treated with 5-fluorouracil. D) Colon mucosa of the group treated with 2.5 mg/kg copper (II) complex. E) Colon mucosa of the group treated with 5 mg/kg copper (II) complex. Rat colonic tissue was stained with methylene blue. Magnification: 20x.
(TIF)

Figure S2 **Histological study of colon cancer in rats.** A) Normal colon mucosa. B) Colon mucosa of the group exposed to AOM.C) Colon mucosa of the group treated with 5-fluorouracil. D) Colon mucosa of the group treated with 2.5 mg/kg copper (II) complex. E) Colon mucosa of the group treated with 5 mg/kg copper (II) complex. The sections were cut parallel to the muscle layer. H & E staining, 100× magnification.
(TIF)
